# Magnetic Resonance Imaging Assessment of Fatigue Injury during Exercise

This article has been retracted.

**DOI:** 10.1155/2022/9971966

**Published:** 2022-06-16

**Authors:** Zhengguo Ai, Na Li, Jing An, Lei Zhang

**Affiliations:** ^1^School of Sport Economics and Management, Tianjin University of Sport, Tianjin 301617, China; ^2^School of Sport, Daqing Normal University, Daqing, Heilongjiang 163712, China; ^3^Daqing Oilfield General Hospital, Daqing, Heilongjiang 163700, China; ^4^Section of Recruitment and Employment, Harbin Sport University, Harbin, Heilongjiang 150008, China; ^5^Department of Physical Education, Heilongjiang Institute of Technology, Harbin, Heilongjiang 150050, China

## Abstract

In order to investigate the changes of temporal function metabolism of lumbar and back muscles after exercise, a magnetic resonance imaging- (MRI-) based assessment of fatigue injury during exercise was proposed. A total of 100 healthy adult volunteers were selected, including 48 males and 52 females, aged from 19 to 30 years, with an average age of 24.8 + 2.3 years. They were divided into four groups according to the different time points of 0, 15, 30, and 45 minutes after exercise, with 25 persons in each group. PHILIPS Achieva 3.0 T Tx MRI scanner was used to perform BOLD and T2-mapping before and after exercise in four groups of healthy volunteers. All data were analyzed by statistical software. The results showed that the total CSA of the dorsi extensor muscle group and the CSA value of the dorsi extensor muscle group at different levels at different time points before and after exercise increased slowly in exercise period and decreased rapidly in recovery period. It was verified that BOLD MRI and T2-mapping imaging can indirectly evaluate the trend of CSA water metabolism and blood oxygen level in healthy adults after exercise.

## 1. Introduction

The lumbar dorsiflexors, including the multifidus longissimus and iliocostus muscles, are the most important part of the core muscles of the human body. Its main role is to participate in the bearing of the spine to maintain human standing posture to maintain the shape of the spine and participate in human walking and other activities. The extensor dorsi muscle group is the largest at the lumbar level, but it is also the most vulnerable part [1]. Long-term poor posture or bending weight can make the low back muscle group (mainly multifidus erector longissimus) in passive stretch or contraction state for a long time. This can lead to insufficient oxygen supply to local muscle tissue, accumulation of metabolites, and stimulate local formation of injurious aseptic inflammation. Severe cases can cause local soft tissue hyperplasia, adhesion, and even degeneration. Patients show recurrent lumbar pain or discomfort, which is often clinically diagnosed as lumbar muscle strain or chronic lower backpain (LBP) [2]. At present, the diagnosis of psoas muscle strain or LBP patients mainly depends on the signs and symptoms, and its treatment is mostly rehabilitation training or massage acupuncture laser irradiation. At present, imaging evaluation of the paralumbar muscles in these patients is only limited to morphological evaluation, including measurement of muscle CSA and CT value of lumbar and back muscles to evaluate the degree of muscle atrophy and fat infiltration.

## 2. Literature Review

Wouters et al. found that long-term poor posture or bending and loading can keep the low back muscles (mainly the multifidus erector longissimus) in a passive stretch or contraction state for a long time. This will lead to insufficient oxygen supply to local muscle tissue, accumulation of metabolites, and stimulate local formation of injurious aseptic inflammation. Severe cases can cause local soft tissue hyperplasia, adhesion, and even degeneration. Patients show recurrent lumbar pain or discomfort, which is often clinically diagnosed as lumbar muscle strain or chronic lower backpain (LBP). At present, the diagnosis of psoas muscle strain or LBP patients mainly depends on the signs and symptoms, and its treatment is mostly rehabilitation training or massage acupuncture laser irradiation [3]. Zhang et al. found that imaging assessment of the paralumbar muscles in these patients is currently limited to morphological assessment, including measurement of muscle CSA and lumbar back muscle CT values to assess muscle atrophy and fat infiltration [4]. Zhu et al. believed that BOLD MRI could achieve noninvasive detection of microdeoxygenated hemoglobin changes in tissues and could be superimposed with high-resolution anatomical images. Therefore, BOLD MRI could not only achieve accurate spatial positioning but also noninvasive reaction of microblood perfusion in tissues. T2-mapping is a magnetic resonance examination technology that uses T2 relaxation time as a measurement index to quantitatively analyze changes in tissue components. It can also achieve accurate spatial positioning and detect changes in microwater content in soft tissues [5]. Studies have proved that BOLD MRI and T2-mapping can be applied to muscle functional magnetic resonance imaging. Therefore, this study intends to use functional magnetic resonance BOLD MRI and T2-mapping to scan the lumbar extensor muscle group before and after exercise in healthy young people, as shown in Figure 1. Observe the changes of R2^∗^ and T2 values of the lumbar dorsiflexor muscle group before and after exercise. Tantawy et al. analyzed the characteristics of blood perfusion changes of the lumbar dorsi muscle group and water molecule changes in muscle space before and after exercise and compared with the changes of muscle cross-sectional area before and after exercise, to further explore the feasibility of functional magnetic resonance assessment of lumbar and back muscle function [6].

## 3. Methods

In order to further clarify its curative effect and therapeutic advantage, medical records were retrospectively analyzed to explore the clinical effect of magnetic resonance imaging on fatigue injury caused by exercise. A total of 100 healthy volunteers were selected, including 48 males and 52 females, aged from 20 to 28 years, with an average age of (24.8 + 2.3) years. The average body weight was (57.52 kg ± 9.20 kg). The average height is (164.28 + 7.26) cm. The body mass index is 17.78~ 23.65 kg/m^2^, and average body mass index is (20.77 ± 2.26) kg/m^2^. All volunteers were scanned before exercise and divided into four groups with 25 participants in each group, including 12 males and 13 females, according to different time points of 0, 15, 30, and 45 minutes after exercise.

If skeletal muscle's own blood perfusion and water molecular content are affected, the results of the study will produce errors [7]. The content of muscle fiber in the skeletal muscle and the activity of the target muscle before the experiment will affect the experimental results. Muscle degeneration caused by any disease through special muscle resistance training or heavy manual labor will lead to changes in the content of muscle fibers in the skeletal muscle compared to normal people, as well as changes in the amount of blood perfusion in the skeletal muscle. However, the intense activity of the target muscle group before the examination will increase the content of water molecules in the intracellular and intercellular space of the skeletal muscle, thus interfering with the experimental results [8]. Therefore, the selection criteria for volunteers are listed below:

1. Normal serial MRI scans of healthy adult volunteers showed no abnormalities in lumbar and paravertebral muscles
2. Light manual workers, such as student civil servants
3. Within 48 hours before the scanning, the volunteers had not done strenuous exercise such as running, playing ball, fitness, and swimming
4. Fasting within 2 hours prior to scanning and coffee drinking within 24 hours prior to scanning

The exclusion criteria for volunteers are as follows:

1. Routine magnetic resonance sequence lumbar degenerative changes: bulging of lumbar intervertebral disc or atrophy of lumbar muscle and fat infiltration
2. People who have undergone special resistance training of lumbar and back muscles and heavy manual workers, such as athletes and fitness coaches
3. Low back pain, long-term bed rest, low back surgery, history of scoliosis deformity, neuromuscular diseases, etc.
4. Unable to complete the lumbar muscle training program
5. The volunteers could not undergo MRI tests for claustrophobia or carrying metal objects

A Dutch PHILIPS Achieva 3.0 T superconducting magnetic resonance scanner (maximum gradient field intensity > 80 Mtm, maximum gradient switching rate 220 mT (m)) was used. The acquisition coil was an orthogonal 15-channel spinal coil. The scanning flow chart is shown in Figure 2. Then, with the lumbar spine as the axis, sagittal T2WI scan was performed with 9 layers and a thickness of 0.4 mm.

Axial T1WI scanning was performed with sagittal T2WI as the reference plane and the upper edge of L3 and L4 as the center. The scanning layers were 32, and the interval was 0.4 mm. All volunteers underwent preexercise scanning and were divided into 4 subgroups according to time points: 0 min, 15 min, 30 min, and 45 min. Each subgroup underwent scanning at corresponding time points. Scan sequence and parameters are shown in Table 1 [9].

The whole exercise process was guided by a special person and lasted for about 10 minutes. After 15, 30, and 45 minutes of exercise, the volunteers lay flat on a simple folding bed and rested until the scan to avoid the influence of paravertebral muscle tension caused by standing or sitting position.

Precautions before scanning were as follows: the volunteers rested for 30 minutes before scanning, lying flat on a simple folding bed. Before scanning, the volunteers used a double abdominal band to compress the abdomen to avoid artifacts caused by excessive breathing. The volunteers lay flat on the scanning bed with their heads fixed. In order to prevent discomfort caused by the noise during the scanning, they wore earphones to reduce the noise. Foam boards were placed below the waist, and foam pads were placed on both lower limbs to raise the legs, so as to reduce the gap between the waist and the scanning bed. At the same time, volunteers were asked to adopt chest breathing as far as possible during the scanning process, so as to reduce the generation of respiratory motion artifacts [10]. During the scan, place your hands in front of your chest, but avoid crossing them. Keep your elbows out of your body and as far away from your waist as possible to minimize artifacts. If the volunteers were female, they should remove their underwear to avoid metal artifacts. They were asked to keep their bodies still during the scanning and avoid motion artifacts [11]. The exercise method is as follows: adopt simple Roman stool to do goat stand up movement, namely, the upper body antigravity flexion and extension movement. In the past, dorsiflexion was a movement, the whole movement process was divided into three groups, each group did 15 movements, and the interval between groups rested for 30 seconds. The main points of action are as follows: the feet are fixed, the body lies on the bench, the upper body slides to the lower abdomen and sticks to the side of the stool, the hands are crossed in front of the chest when the action is carried out, the upper body is quite upward as far as possible, when the highest point stops for three seconds, and then the body overcomes the gravity effect and slowly goes down [12]. The whole movement should be maintained in the way of fast rise and slow fall, not relying on gravity or inertia to complete the action quickly.

After scanning, GE ADW4.4 postprocessing workstation was used for image processing and analysis. Taking the upper edge of L3 and L4 vertebrae as the level of interest, the boundary of longissimus multifidus and iliocostus muscle was delineated in the cross-section of the corresponding level, and the CSA and corresponding T2 values of each muscle were recorded. The R2^∗^ values of each muscle were measured by the same method. During the measurement of muscle values, the range of the region of interest should avoid tendon and intramuscular fat components. The postprocessing threshold of BOLD MRI is 71~ 201, the confidence is 0.05, and the color level is 20~ 100. The postprocessing threshold of T2-mapping was 10, the confidence was 0.05, the value of color levels ranging from 33 to 71 was measured by two attending physicians who had been engaged in bone and muscle imaging diagnosis for a long time by the double-blind method, and the average value was calculated [13].

SPSS 24.0 software was used for statistical analysis of the general condition of the volunteers (height, weight, age, BMI) and independent sample *t*-test. One-way ANOVA was used for the CSA, T2 values, and R2^∗^ of all muscles of different genders (longissimus multifidus and iliocostal muscle) on the left and right sides at multiple time points before and after exercise. The LSD method was used for pairwise comparison of CSA, T2 values, and R2^∗^ values of all muscles. Pearson correlation analysis was used for correlation analysis.

The general information of male and female healthy volunteers is shown in Table 2. After statistical analysis, the average height and weight of male were higher than that of female (*P* < 0.05), while there were no significant differences in age and body mass index (BMI) between male and female (*P* > 0.05).

The general situation of volunteers in each group was shown in Table 3. After statistical analysis, there was no significant difference in the height, weight, age, and BMI of volunteers in each group (*P* > 0.05).

The comparison of the total CSA of the dorsi extensor muscle group at different time points before and after exercise showed that the changes of the total CSA of the dorsi extensor muscle group at different time points before and after exercise were statistically significant (*P* < 0.05). CSA increased 15 minutes after exercise compared with 0 minutes before exercise and decreased 30 and 45 minutes after exercise compared with 15 minutes after exercise. There is a comparison of CSA of dorsi extensor muscle groups at different levels at different time points before and after exercise by statistical analysis, L3 upper margin layer, and L4. The changes of CSA of the dorsi extensor muscle group at the upper margin were statistically significant at different time points before and after exercise (*P* < 0.05). CSA increased 15, 30, and 45 minutes after exercise compared with that before exercise, and CSA increased 15, 30, and 45 minutes after exercise compared with that at 0 minutes after exercise [14].

The comparison of CSA of muscles at different levels at different time points before and after exercise was shown in Figure 3. After statistical analysis, THE CSA of multifidus muscle at L4 level increased 15 and 45 minutes after exercise compared with before exercise and decreased 30 minutes after exercise compared with 15 minutes after exercise, with statistical significance (*P* < 0.05). The CSA of multifidus muscle at L3 increased 15 minutes after exercise compared with before exercise and decreased 30 minutes after exercise compared with 15 minutes after exercise, with statistical significance (*P* < 0.05). The CSA of the longissimus muscle at L4 increased 15, 30, and 45 minutes after exercise compared with that before exercise, and the CSA increased 15, 30, and 45 minutes after exercise compared with that at 0 minutes after exercise with statistical significance (*P* < 0.05). L3 level of longissimus muscle increased 15 minutes after exercise compared with 0 minutes before exercise and decreased 30 and 45 minutes after exercise compared with 15 minutes after exercise, with statistical significance (*P* < 0.05).

CSA changes of iliocostal muscle at L3 and L4 levels at different time points before and after exercise were not statistically significant (*P* > 0.05).

The comparison of the CSA of the left and right muscles at different levels at different time points before and after exercise showed that the CSA at L4 level increased 15 and 45 minutes after exercise compared with before exercise and decreased 30 minutes after exercise compared with 15 minutes after exercise, with statistical significance (*P* < 0.05). At L3 level, the CSA of the left multifidus muscle increased 15 and 45 minutes after exercise compared with before exercise, decreased 30 minutes after exercise compared with 15 minutes after exercise and increased 45 minutes after exercise compared with 30 minutes after exercise, with statistical significance (*P* < 0.05). The CSA of the right longissimus muscle at L4 level increased 15, 30, and 45 minutes after exercise compared with that before exercise, the CSA at L4 level increased 15, 30 and 45 minutes after exercise compared with that at 0 minutes after exercise, and the difference was statistically significant (*P* < 0.05). CSA increased in 45 minutes compared with 0 minutes after exercise, and the difference was statistically significant (*P* < 0.05). At L3 level, the CSA of bilateral longissimus muscle increased 15 minutes after exercise compared with 0 minutes before exercise and decreased 30 and 45 minutes after exercise compared with 15 minutes after exercise, and the differences were statistically significant (*P* < 0.05). There was no significant difference in CSA at L3 and L4 levels at different time points before and after exercise of bilateral iliocostal muscles (*P* > 0.05).

The comparison of CSA of left and right muscles at different levels and different genders at different time points before and after exercise was statistically analyzed. In male volunteers, the CSA at L4 level increased 15 minutes after exercise compared with before exercise, CSA decreased 30 minutes after exercise compared with 15 minutes after exercise, and CSA increased 45 minutes after exercise compared with 30 minutes after exercise, with statistical significance (*P* < 0.05). At L3 level, the CSA of right multifidus muscle increased 15 minutes after exercise compared with before exercise, increased 15 minutes after exercise compared with 0 minutes after exercise, and decreased 30 minutes after exercise compared with 15 minutes after exercise, with statistical significance (*P* < 0.05). The CSA of right multimultius muscle of female volunteers increased 15, 30, and 45 minutes after exercise compared with that before exercise and 45 minutes after exercise compared with that 0 minutes after exercise, with statistical significance (*P* < 0.05). The CSA of left multifidus muscle at L4 level increased 30 and 45 minutes after exercise compared with that before exercise, and the difference was statistically significant (*P* < 0.05). L3 level CSA of right multifidus muscle increased at 0 min after exercise compared with before exercise and decreased at 15, 30, and 45 min after exercise compared with 0 min after exercise, and the difference was statistically significant (*P* < 0.05). L3 level CSA of left multifidus muscle increased 15 minutes after exercise compared with before exercise and decreased 30 minutes after exercise compared with 1S after exercise, with statistical significance (*P* < 0.05) [15, 16].

## 4. Discussion

The lower part of the human dorsi extensor muscle group starts from the posterior edge of the dorsal iliac ridge of the sacrum and passes up to the level of the L4 vertebra to the longissimus multifidus and iliocostus muscles. The iliac costal muscle is located in the inner side of the posterior edge of each costal arch, and its main function is to participate in spinal dorsi extension and assist the rotation of the upper body. The longissimus is attached upward to the mastoid process, and the multifidus arises laterally in the form of a short tendon of lumbar vertebrae's nipple. At the top, the spinous process of the upper vertebral body, the longissimus muscle, and the multifidus muscle are mainly involved in spinal dorsi extension [17, 18]. The dorsiflexor muscle group is the most important part of the core muscle group of the human body, and its role is to maintain the normal shape of the spine and participate in the maintenance of walking and posture. The dorsi extensor muscle group is the largest at the level of lumbar vertebrae, its morphology and structure are relatively complex, and it is also the most vulnerable to injury. It is closely related to LBP strain of psoas muscle or disc herniation, and it is the most important muscle group to be paid attention to in clinical rehabilitation training. MRI has a high resolution of soft tissue, and its display of the lumbar extensor muscle group is superior to CT and ultrasound and with the advent of functional MRI. In particular, magnetic resonance phosphorus spectrum analysis can not only observe the changes of CSA before and after muscle exercise but also dynamically monitor the mutual transformation process between phosphocreatine and ATP before and after muscle exercise. However, phosphorus spectrum analysis requires special magnetic resonance detection equipment and is difficult to be popularized in clinical use. Bold MRI is widely used in the study of nervous system function, usually to detect changes in local blood M flow in the brain under a certain disease state or a certain task state, so as to reflect the range of lesions or functional areas in the brain. With the development of fMRI, BOLD MRI has also been gradually applied to the research outside the nervous system, including kidney, liver, and skin tissue. However, BOLD MRI is rarely reported in the study of the skeletal muscle system, especially in the study of the lumbar dorsi muscle group [19, 20]. In the 1990s, Ogawa et al. discovered that deoxygenated hemoglobin changed the signal of blood vessels and surrounding water molecules, and this changed signal could be detected by gradient echo sequence of high-field MRI, thus discovering BOLD enhancement effect. Deoxyhemoglobin in the human body is a paramagnetic material, and its iron ions contain four unpaired electrons; so, it can affect the relaxation time of neighboring protons. When the amount of deoxygenated hemoglobin in a single blood vessel increases, decreased T2 or T2^∗^ signaling of water molecules in and around blood vessels, that is, the transverse relaxation rate of adjacent water molecules R2 (1/T2)和R2^∗^ (1/T2^∗^) is increased. The decrease of R2^∗^ signal in tissues can indirectly reflect the decrease of deoxygenated hemoglobin content in small blood vessels in tissues, thus reflecting the changes of blood perfusion volume in tissues in the resting task state.

There were significant differences in R2^∗^ values of the left and right iliocostal muscles at the L3 upper margin of normal healthy volunteers before and after exercise, and the difference was more significant in the female group (left change > right) but not in the male group. Comparison of the CSA of the left and right iliocostal muscles at the L3 upper margin before and after exercise showed that the CSA changes of the left iliocostal muscles before and after exercise were more obvious in the female group than in the right side, while the difference between the left and right sides was not obvious in the normal male group. However, there was no significant difference in the changes of CSA or R2^∗^ before and after muscle exercise at the upper edge of L4 in both male and female groups. After analysis, the R2^∗^ values and CSA changes of the left and right iliac-costal muscles before and after exercise at the upper margin of L3 in the female group were more obvious than those on the right. The two showed corresponding consistency, and the difference existed in the female group, while there was no difference in the male group. The reason may be that during the whole dorsiflexion movement, the longissimus muscle of the female multifidus is not strong enough to contralateral iliocostal muscle contraction, and corresponding blood flow is reduced due to the compensatory assistance of one side (left) iliocostal muscle contraction. In L4, there was no significant difference in CSA and R2^∗^ between the left and right sides before and after the exercise of each muscle in the upper margin layer, but L3. There are significant differences between the left and right iliocostal muscles at the upper margin, which may be due to the fact that the dorsal extensor muscle group at L4 and L3 is mainly involved in the dorsal extension movement, while the iliocostal muscles at L3 are not only involved in the dorsal extension movement but also have the function of assisting lateral rotation.

## 5. Conclusion

BOLD MRI and T2-mapping's imaging can indirectly assess the trend of CSA water metabolism and blood oxygen level in the back muscle of healthy adults after exercise. After exercise, the CSA and T2 values of lumbar and back muscles showed slow movement: rising and rapid downward trend in the recovery period; R2^∗^ showed a rapid decrease in the exercise period and a rapid increase in the recovery period. The T2 value of the longissimus muscle at level 3 increased earlier than that at L4, and the change rate of T2 value of the longissimus muscle at the right level of L3 increased earlier than that at the left level of L3 and L4. The T2 value of the horizontal left iliocostal muscle increased later than the right side of L4. The left and right sides of the muscle could affect the change rate of T2 value of the longissimus muscle and iliocostal muscle after exercise. The CSA of longissimus multifidus of different genders increased slowly during the exercise period and maintained a trend during recovery period in females, while decreased slowly during the recovery period in males. The changes of CSA after exercise of multifidus muscle and longissimus muscle were influenced by different genders.

## Figures and Tables

**Figure 1:** Flow chart of muscle functional magnetic resonance scan.

**Figure 2:** Magnetic resonance scanning flow chart.

**Figure 3:** Comparison of CSA of muscles at different levels at different time points before and after exercise.

**Table 1:** MRI scanning sequence and scanning parameters.

	Scan sequence	Sweeping solid (mm)	Echo time (ms)	Repeat time (ms)	NEX	Thickness of layer (mm)	Interlamellar spacing (mm)	The layer number of scanning
T2WI sagittal view	PSE	0.91 × 1.32 × 4.00	120	2000	2	4	0.4	9
TlWI cross-sectional place	FSE	0.71 × 0.90 × 4 00	7.6	344	3	4	0.4	32
BOLD cross-sectional place	EPI	1.5U × 1.50 × 4.00	3.7/10.3/15.9/21.5/27.1/32.7	466	6	3	0.7	24
T2-napping cross-sectional place	FSE	0.76 × 0.76 × 0.30	7/13/19/25/31/37	1974	1	3	0.7	24

**Table 2:** Male and female volunteers were generally compared.

	Cases	Height (cm)	Weight (kg)	Age (year)	BMI (kg/m^2^)
Male	48	170.75 ± 5.43	63.28 ± 8.31	24.48 ± 2.56	21.72 ± 2.42
Female	52	160.05 ± 4.95	53.17 ± 6.56	23.39 ± 2.06	20.28 ± 2.26
*T* value		11.06	8.45	2.53	3.37
*P* value		<0.001	<0.001	0.054	0.131

**Table 3:** Analysis of general situation among each group.

Time						
	First group	Second group	Third group	Fourth group	*F*	*P*
Height (cm)	165.34 ± 7.25	164.41 ± 8.37	164.72 ± 7.18	165.92 ± 8.14	0.180	0.963
Weight (kg)	56.83 ± 7.54	57.54 ± 7.53	56.38 ± 8.31	57.13 ± 6.89	0.653	0.349
Age (year)	23.3 ± 3.1	23.8 ± 2.0	22.8 ± 1.7	22.7 ± 0.6	0.543	0. 197
BMI (kg/m^2^)	21.3 ± 1.9	21.7 ± 2.9	20.7 ± 2.2	20.4 ± 2.5	1.326	0.078

## Data Availability

The data used to support the findings of this study are available from the corresponding author upon request.
